# An Efficient Machine Learning-Based Feature Optimization Model for the Detection of Dyslexia

**DOI:** 10.1155/2022/8491753

**Published:** 2022-07-09

**Authors:** Nazir Ahmad, Mohammed Burhanur Rehman, Hatim Mohammed El Hassan, Iqrar Ahmad, Mamoon Rashid

**Affiliations:** ^1^Department of Information Systems, Community College, King Khalid University, Abha, Saudi Arabia; ^2^Department of Computer Engineering, Faculty of Science and Technology, Vishwakarma University, Pune, India

## Abstract

Dyslexia is among the most common neurological disorders in children. Detection of dyslexia therefore remains an important pursuit for the research works across various domains which is illustrated by the plethora of work presented in diverse scientific articles. The work presented herein attempted to utilize the potential of a unified gaming test of subjects (dyslexia/controls) in tandem with principal components derived from data to detect dyslexia. The work aims to build a machine learning model for dyslexia detection using comprehensive gaming test data. We have attempted to explore the potential of various kernel functions of the Support Vector Machine (SVM) on different number of principal components to reduce the computational complexity. A detection accuracy of 92% is obtained from the radial basis function with 5 components, and the highest detection accuracy obtained from the radial basis function with 3 components is 93%. On the contrary, the Artificial Neural Network(ANN) shows an added advantage with minimal number of hyperparameters with 3 components for obtaining an accuracy of 95%. The comparison of the proposed method with some of the existing works shows efficacy of this method for dyslexia detection.

## 1. Introduction

One of the most complicated neurological brain disorders that is attracting attention among researchers in modern neuroscience is Dyslexia [1]. The International Dyslexia Association defines dyslexia as a disorder identified by difficulties with spelling, language processing, and accurate word recognition. The overall paradigm of dyslexia can be summarized in Figure 1. The main actors of dyslexia consist of phonological disorder (PD), visual disorder (VD), and auditory disorder (AD). These disorders start to evolve from the time of birth and manifest themselves into an abnormality. The associated abnormality with these actors plays a very critical role in shaping the personality of a person. The consequences are multifold with numerous behavior deficits (BD) and cognitive deficits (CD). Most people think of dyslexia as a disorder in which a person is seeing letters and words backwards such as seeing “*b*” as “*d*” and vice versa, “was” as “saw” and vice versa. However, the truth is that people with dyslexia see things the same way as everyone else. Dyslexia is caused by a phonological processing problem [2] meaning people affected by it have trouble not with seeing language but with manipulating it. For example, if a person with dyslexia hears a word such as “heat” and then someone asks him/her to remove the first word (which is “*h*”). It would be very difficult for a person with dyslexia to tell what word is left (“eat”).

Another example of a person with dyslexia is that they tend to break a word in parts to read it, thus delaying reading comprehension. Dyslexia affects about 5–17% of population across most languages [3]. The dyslexia condition emerges at some stage in childhood and evolves progressively in adolescence. This effect hampers the academic growth and subsequently diminishes self-esteem and confidence [4]. On the other hand, the emergence of transformative healthcare technologies has catalyzed a revolution in provisioning and operational functioning of healthcare services, driven mostly by Computer Aided Detection and Diagnostic systems, interchangeably referred to as CAD systems. Recent advances in imaging technologies have made it plausible for medical practitioners to use advanced and hybrid imaging techniques such as PET, USG, X-Rays, CT scan, fMRI, and SPECT, in addition to others. Enhancements in these techniques enable medical practitioners to gather detailed information about body organs and physiology. These techniques typically make use of internal, external, or both sources of energy [5, 6].

The work proposed herein have multiple advantages that make it a potential candidate as a dyslexia detection framework. This does not consider any imaging modality information for the development of CAD for dyslexia. The information used is generated using a gamified online test structured in such a way that behavioral and cognitive deficits are perceived and quantified. It utilizes acquired data to establish a machine learning framework with principal component analysis. With SVM and ANN as machine learning frameworks, PCA is seen to be very effective in the detection of dyslexia. Moreover, PCA significantly reduces the computational overhead of the model since it has to deal with narrow feature space.

The overall organization of the paper is as follows: section 2 presents some of the existing work in the domain of dyslexia detection. The proposed framework is illustrated in section 3 of the paper, while the experimental setup along with the results are discussed in section 4 of the paper.  Section 5 presents the conclusion of the work.

## 2. Related Work

With the advent of smart devices that are utilized in different domains such as healthcare, business organizations, educational sector, cities, and agriculture, a humongous amount of data is being generated. These insights to these data open new challenges and possibilities in a wide range of applications. The information collected from various sources in a healthcare setup open possibility for early detection or future prediction of various diseases. Studies presented in [7–10] have leveraged the healthcare data for different detection tasks. Studies by [11, 12] reveal that the collection of data sets for dyslexia are relatively cheap when we create a dataset by using standardized psychoeducational tests and learner's handwritings. This is the reason that we are using a gamified online test for the study. So, the use of these data sets actually provides 2 benefits: first is that it is very cheap to collect and the other one being that the size of the data set, that is, in terms of features is very large, which is one of the fundamental requirements for building a stable machine learning model. The next subsection provides a list of machine learning algorithms that have been proposed from time to time for the detection of dyslexia. All these studies have used different types of machine learning algorithms and datasets of varying nature and sizes. The study by [13] demonstrated the application of artificial neuron networks to identify the presence of dyslexia in school children. The study used the test score as the data and MLP architecture of ANN. With a 10-fold cross validation, an accuracy of 75% was reported in the study.

The work presented by [14] used all sequences of machine learning algorithms which include support vector machines, artificial neural networks, and k-means. MRI scans were used to classify between dyslexia and control groups. With a dataset size of 56, ANN showed up with the best accuracy of 94.8%. The work done by [15] demonstrates the use of MRI scans for discriminating dyslexia and control cases. The study is carried out on a dataset of 236 subjects with SVM as the ML algorithm. An accuracy of 83% was reported in this study. EEG scans of 80 subjects were used for the diagnosis of dyslexia at an early stage using machine learning algorithms which included the *k* means, ANN, and fuzzy logic classifier with an average accuracy of 89.6%, 89.7%, and 85.7%, respectively, by [16]. Another study based on EEG scans is presented in [17] on 6 subjects with a median age group of 5. Here, a multilayer perception model was used to detect dyslexia by analyzing brain activity signals, achieving an accuracy of 85%. MATLAB's LIBSVB toolbox was used to implement the linear support vector machine classifier on 61 MRI scans to discriminate a dyslexia biomarker using white matter features of the brain. The accuracy reported in this study for dyslexia detection is 83.6%.

The work done in [18] categorizes dyslexia and nondyslexia cases on MRI scan data of 925 subjects using linear SVM. The study reports an accuracy of 80%. A linguistic computer game-based dyslexia detection was done by [19] on a 267 subject dataset utilizing eye tracker features. This study reports an accuracy of 85% using the SVM from the LIBSVM Toolbox of MATLAB. Another eye tracker-based dyslexia detection was performed by a study carried by [3] on a dataset of 185 subjects. The SVM was used with automatic recursive feature elimination, obtaining an accuracy of 96%. Another study wherein the SVM has been inducted for dyslexia detection on an eye tracking feature is reported in [20–24]. An accuracy of 80% on a dataset size of 97 is achieved in this work.

## 3. Proposed Methodology

The methodology adopted for this study is pictorially shown in Figure 2. With a large number of methodologies existent on the use of imaging modalities for dyslexia detection, the utilization of the gaming-based tests is also being explored for the potential detection methodology for dyslexia. The next subsection discusses the mathematical framework of the work from start

Assuming a feature vector (F_mi_) of each subject, we should see Eq

(1) $$\begin{array}{c} F_{mi}=\left[f_{11},f_{12},\ldots ,f_{mi}\right], \end{array}$$

where *m* corresponds to subject number and *i* corresponds to each index of the feature vector. For the complete feature space in 2D, we should see Eq

(2) $$\begin{array}{c} F_{s}=\left[\begin{array}{ccc} F_{1,1} & F_{1,2\ldots } & F_{1,198}\\ F_{2,1} & F_{2,2\ldots } & F_{\begin{array}{c} 2,198\\ \vdots \\ \vdots \end{array}}\\ \; & \; & \;\\ F_{m,1} & F_{m,2\ldots } & F_{m,198} \end{array}\right],F_{1,1}\;\epsilon \;{\mathbb{R}}^{3644\;X\;196}.\\ \; \end{array}$$

With *F*_*s*_, we estimate an accuracy parameter *A*_*u*_ from a set of machine learning kernel functions corresponding to SVM. In addition, the same accuracy parameter is estimated for the ANN. Having obtained an *A*_*u*_ from a feature space of size 3644 × 196, our aim is to reduce the feature space by weighted reduction for improving *A*_*u*_. To put it in a more generic way, we aim to obtain the best possible *A*_*u*_ with a feature space which maximizes *σ*^2^ for all *F*_*i*,*j*_. Initially, a set of parameters are chosen for different kernel functions of SVM as given in equations (3)–(8)

(3) $$\begin{array}{c} k\left(x,y\right)=\;x^{T}y+c, \end{array}$$

(4) $$\begin{array}{c} k\left(x,y\right)=\exp\;{\left(-\sigma 1\|x-\mathrm{y\|}\right)}^{2}, \end{array}$$

(5) $$\begin{array}{c} k\left(x,y\right)=\exp\left(\frac{-\|x-\mathrm{y\|}}{\sigma 2}\right), \end{array}$$

(6) $$\begin{array}{c} k\left(x,y\right)=\tanh\left(kx.y+c\right), \end{array}$$

(7) $$\begin{array}{c} k\left(x,y\right)=\exp\left(\frac{J_{v+1}\left(\sigma 3\;\|x-\mathrm{y\|}\right)}{\|x-{\mathrm{y\|}}^{-n\left(v+1\right)}}\right), \end{array}$$

(8) $$\begin{array}{c} k\left(x,y\right)=1+xy+xy\min\left(x,y\right)-\frac{x+y}{2}\min{\left(x,y\right)}^{2}+\frac{1}{3}\min{\left(x,y\right)}^{3}. \end{array}$$

These equations correspond to kernel tricks, namely, linear, radial basis function, Laplace, hyperbolic tangent, Bessel, and linear spline, respectively. These 6 kernel functions yield 6 machine learning algorithms whose potential we wish to explore with the change in feature space size. The choice of the kernels as given in eq. 4, eq. 5, and eq. 7 largely depends on the tunable parameters *σ*1, *σ*2,  and *σ*3, respectively. The selection of these 3 parameters determines the efficacy of the kernel in specific and the SVM as a classifier in general. The selection of *σ*1, *σ*2,  and *σ*3 can neither be underestimated nor overestimated. If the values are overestimated, the kernel function will behave more like a linear function and thus losing the capability of a nonlinear projection. On the other hand, if the values are underestimated, the decision boundary will be sensitive to the noisy data; thus, there will be a lack of regularization.

In line with this rationale, the values of *σ*1, *σ*2,  and *σ*3 are set as 0.15. With all these parameters of the kernel function set, we implement principal component analysis on *F*_*s*_ to help us extract a new set of *F*_*s*_ coefficients. The main idea of applying principal component analysis is to reduce the higher dimensionality of a feature space having large correlated data with a lower dimensionality feature space having small correlated data. The principal components derived from the original data tend to capture most of the variance of the data and hence can be effectively utilized to train a classifier model.  Figure 3 shows an instance wherein we have plotted 100 principal components against the amount of variance that they have captured in the form of eigen values. As can be seen in Figure 3, the first few components capture almost all the variance of the data implying its efficacy. Algorithm 1 shows a pseudocode for the proposed methodology.

## 4. Experimental Results

The dataset [1] chosen for this study is a thorough evaluation of the following components of language speaking and understanding: phonological awareness, morphological awareness, visual discrimination and categorization, alphabetic awareness, syllabic awareness, semantic awareness, auditory discrimination and categorization, visual working: memory, and sequential auditory: working memory. The setup is quite contrasting to the setups which use different types of imaging modalities as a tool for detecting dyslexia. The dataset is 3644 subjects, 2 class-labeled data with 196 attributes.  Figure 4 shows the distribution of the cases with respect to various age groups. The number of dyslexic and nondyslexic cases is well distributed in the range of 07 to 17 years.

Figure 5 shows the percentage of dyslexia subjects' age wise. The point to observe here again is that the distribution is almost evenly distributed. With the given feature set, the proposed model uses two classifiers. Several classification methods exist, which include quadratic discriminant analysis (QDA), linear discriminant analysis (LDA), decision trees, maximum entropy classifier, Naive Bayes classifier, K-nearest neighbor, support vector machine (SVM), and Artificial Neural Network (ANN) [18]. The work herein uses the said dataset to detect dyslexia with the SVM and ANN. First, we propose PCA-driven new feature vectors as the indicators for the dyslexia.

Table 1 depicts the dyslexia detection accuracy using 10 principal components. The highest accuracy is achieved by using the radial basis kernel function with a hyperparameter value *σ*1 = 0.5. The lowest detection accuracy is obtained using the spline kernel function for the SVM. Similarly, Table 2 gives a comparative detection accuracy of the 6 kernel functions with 5 principal components: PC1, PC2, PC3, PC4, and PC5. As expected, the accuracies obtained are slightly better compared to the results obtained in Table 2. The reason that can be attributed to this is depicted in Figure 3 wherein it is seen that lower principal components capture most of the variance in the data. The dyslexia accuracy is seen to improve further when the number of components used in the framework of SVM kernels is reduced to 3. The same is depicted in Table 3.

In comparison to a detection accuracy of 92% obtained from the radial basis function with 5 components, the highest detection accuracy obtained from the radial basis function with 3 components is 93%. The capability of principal components in detecting dyslexia is also depicted by the score plot shown in Figure 6. The plot shows how dyslexic and nondyslexic cases are segregated by the two principal components. Firstly, the PC1 shown as the dotted red vertical line divides all the given cases in the direction of the maximum variance. The number of outliers on the application of the first principal component is significantly large. The second principal component as shown in the purple dotted horizontal line is now seen to reduce the number of outliers.

The same methodology for predicting dyslexia using the online gaming-based test is carried out using ANN. The aim of this part of the study was to observe an accuracy improvement by changing the input size of the ANN. We choose a fixed hidden layer size of 10. With two output classes, dyslexic and nondyslexic, the input to the ANN was changed as per the number of principal components retained from the feature space.  Table 4 shows the number of weights learnt by each NN with the changing number of inputs. On one side, the smaller number of components hide most of the information from the data, and on the other hand, the number of components leads to a smaller number of weights that were needed to be learnt. The comparison of the proposed methodology with some of the recent works reported in [15, 25, 26] is tabulated in Table 5. Most of the work reported for the detection of dyslexia has 4 main parameters, namely, the size of the dataset, the nature of the dataset, underlying machine learning approach, and the performance of the overall methodology. Based on these 4 parameters tabulated in Table 5, most of the work has been carried out on a relatively small-sized dataset. The demerit of the small-sized dataset in the machine learning framework is that it lacks generalization. The proposed work is carried out on a dataset which is comparatively much larger than the other reported works and hence is better in terms of generalization.

## 5. Conclusion

As the numbers state, dyslexia is listed over a population of 10% across the globe with consequences from moderate to severe personality changes. In Saudi Arabia, the incidence rate of dyslexia is found to be around 7%. Early detection of this disorder can help effective treatment in most of the cases. With researchers, clinicians and experts from various domains taking a stride to address this issue, the success is not that far away. Artificial intelligence and machine learning in contention with the medical imaging modalities have come up with possibilities of hope. The work presented herein successfully attempted to use an online gaming test-based strategy for the detection of dyslexia. It is pertinent to mention that with the age and lifestyle of the subjects under consideration, online gaming methodology for data acquisition becomes one of the first choices. The work extends by utilizing this acquired data to establish a machine learning framework with principal component analysis. With SVM and ANN as machine learning frameworks, PCA is seen to be very effective in the detection of dyslexia. Moreover, PCA significantly reduces the computational overhead of the model since it has to deal with narrow feature space. The work herein reports an accuracy of 95% with PCA and ANN with nearly 4000 subjects in the overall experimentation setup. The proposed work shows potential as depicted by the comparison of this methodology with some of the existing works. This work can be a promising candidate for the development of the learning management system for dyslexia. In future, the authors will try to improve the results of this research work by employing a deep learning model where optimization will be carried out on input images directly [27, 28].

## Figures and Tables

**Figure 1:** Various actors and consequences in the dyslexia timeline.

**Figure 2:** Framework for PCA-optimized dyslexia detection.

**Figure 3:** Various principal components of the dyslexia dataset versus eigen values.

**Figure 4:** Case distribution against various age groups.

**Figure 5:** Age-wise percentage of dyslexia.

**Figure 6:** Classification of dyslexic and nondyslexic cases by PC1 and PC2.

**Algorithm 1:** Pseudocode of the proposed methodology.

**Table 1:** *A*_u_ with various kernel functions using 10 components.

Kernel functions	Accuracy (*A*_u_)
Linear	89.8
Hyperbolic tangent	81.8
Laplacian (sigma= 0.15)	89.2
Bessel (sigma= 1, degree= 1)	87.4
Spline	80.8
Radial basis (sigma= 0.15)	89.9

**Table 2:** *A*_u_ with various kernel functions using 5 components.

Kernel functions	Accuracy (*A*_u_)
Linear	91.5
Hyperbolic tangent	84.7
Laplacian (sigma= 0.15)	91.5
Bessel (sigma= 1, degree= 1)	91.5
Spline	91
Radial basis (sigma= 0.15)	92

**Table 3:** *A* _u_ with various kernel functions using 3 components.

Kernel functions	Accuracy (*A*_u_)
Linear	93
Hyperbolic tangent	90
Laplacian (sigma= 0.15)	93
Bessel (sigma= 1, degree= 1)	93
Spline	91
Radial basis (sigma= 0.15)	93

**Table 4:** *A* _u_ with various PCs and number of weights learnt.

Principal components inputs to NN	Total weights learnt	Accuracy (*A*_u_)
10	251	89
7	181	89
4	125	91
3	104	95

**Table 5:** Comparison of proposed methodology with various dyslexia detection techniques with state-of-the-art.

Reference	ML technique used	No. of subjects	Accuracy (%)
[21]	SVM	185	90
[22]	SVM	236	65
[23]	SVM	61	83
[11]	ANN	—	75
[20]	Naive Bayes classifier	313	80.1
[24]	Linear discriminate analysis	313	73.9
Proposed	PCA + ANN	3644	95

## Data Availability

Data used in this article will be shared on request to the corresponding author.

## References

[1] Elnakib A., Soliman A., Nitzken M., Casanova M. F., El-Baz G., El Baz A. (2014). Magnetic resonance imaging findings for dyslexia: a review. *Journal of Biomedical Nanotechnology*.

[2] Fletcher J. M., Lyonm G. R., Barnes M., Bradley R., Danielson L., Hallahan D. P. Classification of learning disabilities: an evidence based evaluation.

[3] Tamboer P., Vorst H. C. M., Ghebreab S., Scholte H. S. (2016). Machine learning and dyslexia: classification of individual structural neuro-imaging scans of students with and without dyslexia. *NeuroImage: Clinica*.

[4] Wajuihian S. O. (2012). Neurobiology of developmental dyslexia Part 1: a review of evidence from autopsy and structural neuro-imaging studies. *Optometry Vis Develop, space*.

[5] Barrett H., Swindell W. (1981). Radiological Imaging: The Theory of Image Formation. *Academic Press*.

[6] Bushberg J. T., Seibert J. A., Leidholdt E. M., Boone J. M. (2002). *The Essentials of Medical Imaging*.

[7] Hasan M. K., Ghazal T. M., Ali A. (2021). Linear Discrimination and Quadratic Discrimination Analysisâ€“Based Data Mining Technique for Internet of Things Framework for Healthcare”. *Frontiers in Public Health*.

[8] Ghazal T. M., Anam M., Kamrul Hasan M. (2021). Hep-pred: hepatitis c staging prediction using fine Gaussian svm. *Computers, Materials & Continua*.

[9] Naseer A., Yasir T., Azhar A., Shakeel T., Zafar K. (2021). Computer-aided brain tumor diagnosis: performance evaluation of deep learner CNN using augmented brain MRI. *International Journal of Biomedical Imaging Hindawi-*.

[10] Rizwan M., Shabbir A., Javed A. R., Shabbir M., Baker T., Al-Jumeily Obe D. (2022). Brain tumor and glioma grade classification using Gaussian convolutional neural network. *IEEE Access*.

[11] Rello L., Baeza-Yates R., Ali A., Bigham J. P., Serra M. (2020). Predicting risk of dyslexia with an online gamified test. *PLoS One*.

[12] Sharma P., Kaur M. (2013). Classification in pattern recognition: a review. *International Journal of Advanced Research in Computer Science and Software Engineering*.

[13] Spoon K., Crandall D., Siek K. Towards detecting Dyslexia in children’s handwriting using neural networks.

[14] Spoon K., Siek K., Crandall D., Fillmore M. Can we (and should we) use AI to detect Dyslexia in children’s handwriting?.

[15] Kohli M., Prasad T. V. Identifying dyslexic students by using artificial neural networks.

[16] García Chimeno Y., García Zapirain B., Fernandez-Ruanova B., Saralegui Prieto I. (2014). Automatic classification of dyslexic children by applying machine learning to fMRI images. *Bio-Medical Materials and Engineering*.

[17] Płoński P., Gradkowski W., Marchewka A., Jednoróg K., Bogorodzki P. Dealing with the heterogeneous multi-site neuroimaging data sets: a discrimination study of children dyslexia.

[18] Al-Barhamtoshy H. M., Motaweh D. M. Diagnosis of Dyslexia using computation analysis.

[19] Karim I., Abdul W., Kamaruddin N. Classification of Dyslexic and normal children during resting condition using KDE and MLP.

[20] Benfatto M. N., Seimyr G., Ygge J., Pansell T., Rydberg A. (2016). Screening for dyslexia using eye tracking during reading. *PLoS One*.

[21] Talwani S., Alhazmi K., Singla J., Alyamani H. J., Bashir A. K. (2021). Allocation and migration of virtual machines using machine learning. *Computers, Materials & Continua- Tech Science*.

[22] Sundararajan K., Garg L., Srinivasan K. (April 2021). A contemporary review on drought modeling using machine learning approaches”, computer Modeling in engineering & sciences. *Tech Science*.

[23] Hemant G., Awais M., Bashir A. K. (2022). AI-enabled radiologist in the loop: novel AI-based framework to augment radiologist performance for COVID-19 chest CT medical image annotation and classification from pneumonia. *Neural Computing and Applications*.

[24] Usman M., Lateef O., ChandrenMuniyandi R., Omar K., Mohamad M. (2021). Advance Machine Learning Methods for Dyslexia Biomarker Detection: A Review of Implementation Details and Challenges. *IEEE Access*.

[25] Jothi Prabha A., Bhargavi R. (2019). Prediction of Dyslexia from eye movements using machine learning. *IETE Journal of Research*.

[26] Lakretz Y., Chechik G., Friedmann N., Rosen-Zvi M. ‘Probabilistic graphical models of Dyslexia.

[27] Płoński P., Gradkowski W., Altarelli I. (2017). multi-parameter machine learning approach to the neuroanatomical basis of developmental dyslexia. *Human Brain Mapping*.

[28] Cui Z., Xia Z., Su M., Shu H., Gong G. (2016). Disrupted white matter connectivity underlying developmental dyslexia: a machine learning approach. *Human Brain Mapping*.

